RETRACTED

# Comparative Analysis of Dynamic Characteristics between Electronic Signature and Conventional Signature Based on Computer Vision Technology

**DOI:** 10.1155/2022/4965908

**Published:** 2022-06-26

**Authors:** Chao Feng, Zhongyuan Ji, Jin Zhang

**Affiliations:** ^1^College of Criminal Justice, Shandong University of Political Science and Law, Jinan, Shandong 250014, China; ^2^College of Electronic and Information Engineering, Nanjing University of Aeronautics and Astronautics, Nanjing, Jiangsu 211106, China; ^3^Police Officer Academy, Shandong University of Political Science and Law, Jinan, Shandong 250014, China

## Abstract

During the last two or three decades where innovations in technology have been dominant, especially the rapid development of electronic information technology, various types of electronic devices have been developed for different application areas. It is this technological-assisted equipment that has drastic effects on the lifestyle of every creature in general and human beings in particular. In addition to the other activities or services, technology has enabled human beings to write on electronic devices, which is due to the fact that these devices will generate electronic signature handwriting that is extremely useful for human beings. They may effectively cope with the electronization of traditional signature handwriting and ease the difficulties of authenticating the identification information of the signatory of electronic documents when used in conjunction with electronic documents. This method is frequently utilized in e-government, e-commerce, banking and insurance, medical care, and other industries. This study uses the current mainstream computer vision technology to compare and analyze the handwriting dynamic characteristics of electronic signature and conventional signature. It uses the electronic signature God and software to collect and extract the original characteristic data of user's electronic signature and then extracts the characteristics of average writing speed, duration, and average pressure on the basis of these data for analysis. Among these techniques, the writing time of electronic signature is longer than that of conventional signature, and the average speed of conventional signature notes is higher than that of electronic signature, and when analyzing the average pressure characteristics, the conventional signature pressure is greater than the electronic signature pressure.

## 1. Introduction

At present, electronic signature is widely used in various industries, and its typical representatives are banking, finance, insurance, and other fields. Electronic signatures are separate from digital signatures, which are a cryptographic mechanism that is frequently used to implement electronic signatures. While an electronic signature can be as simple as a name in an electronic document, digital signatures are increasingly being utilized in e-commerce and regulatory filings to implement electronic signatures in a cryptographically secure manner. An electronic signature, also known as an e-signature, is data that is logically linked to other data and utilized by the signatory to sign the linked data. As long as it complies with the requirements of the specific regulation under which it was established, this sort of signature has the same legal standing as a handwritten signature. Due to its wide range of use, some people began to question the difference between electronic signature track and conventional signature track, so as to avoid unnecessary impact caused by large difference between electronic signature and conventional track [1]. Therefore, this study uses computer vision technology to compare and analyze the dynamic characteristics of electronic signature and conventional signature, so as to judge the difference between them [2]. As a new type of handwriting, electronic handwriting is a way for people to form electronic signature handwriting on the equipment by using electronic touch pen. It is a way to express writing activities by digital way. According to the analysis of electronic signature handwriting data structure, its components include electronic image information and electronic data information. Comparing the handwriting of ordinary signature with that of electronic signature, there will be differences in the handwriting written by the same person, which can directly reflect their writing habits and writing pressure.

RETRACTED

Main contributions of this manuscript are as given as follows:

1. Initially, we have focused on how to compare the dynamic characteristics of both electronic and conventional signatures handwriting from the perspective of computer vision technology, which is the main contribution of this study. Likewise, as described in the video tracking algorithm, motion modeling and tracking algorithm, the above algorithm is applied to analyze the dynamic characteristics of electronic signature and conventional signature handwriting.
2. To evaluate the acquired original data of electronic signature and traditional signature handwriting, Wacom electronic signature equipment and analytic software were chosen. The features of writing duration, average speed, and average pressure are examined using computer vision technology, and the dynamic properties of electronic signature and standard signature handwriting are compared.

The remainder of this study is organized as follows.

RETRACTED

In the subsequent section, a detailed and thorough review of the possible literature contents is reported, which is followed by the proposed methodology especially computer vision-based applications. In Section 4, dynamic characteristics of electronic signature and conventional signature handwriting based on computer visual technology have been described, which is followed by results and discussion. Finally, a summary of the study is provided.

## 2. Related Works

At present, many experts at home and abroad have studied the difference between the characteristics of electronic signature handwriting and ordinary signature handwriting. When studying the dynamic characteristics, the parameter changes of handwriting formation stage speed, time length, pressure, and acceleration are analyzed [3]. Font size and writing speed are the most easily changed qualities, according to American academic LEEM et al., but other scholars claim that font collection characteristics, size characteristics, and line characteristics change the most. These metrics are the vital metrics as far as electronic signatures are being concerned. Moreover, if values of these factors are not collected according to the available guidelines, then it is high likely that the developed system has issues [4]. Maksimov combined time dynamic warping (DTW) and variance to conduct a comparative study on the signature duration of standard sitting posture and special sitting posture. The results show that the change of personal writing habits and signature duration will affect the writing posture [5]. Safonova and Safonava research points out that writing on the horizontal plane can maintain stable dynamic characteristics no matter how to adjust the sitting posture [6]. Bakhteev, combined with analysis of variance, compared the average speed, duration, average speed, average pressure, and acceleration of natural signature and *t* camouflage signature. The comparison shows that this feature is very different, which is directly related to the handwriting writing mode of natural signature [7]. Ma uses spectrum analysis, data analysis, and template matching analysis to study the differences in the acceleration, average speed, and pressure changes of the signature pen and imitation handwriting [8]. Ghadhban et al., combined with analysis of variance, compared the pen lifting times and median on the average pressure of handwriting between copy signature and imitation signature. The results showed that there was a significant average pressure difference between the two. At the same time, stroke complexity, signature handwriting size, and handwriting recognition affected the average pressure [9]. By combining nonparametric test and *t*-test, Setyawati selected the ratio between the standard deviation and the average value of data such as writing time, handwriting peak speed, and pressure as the judgment basis. The results showed that there were significant errors in the pressure, speed, and value linearity of imitation signature and imitation signature [10]. Based on the analysis of Dwinata, combined with generalized linear model, it is concluded that there are great differences in writing size, duration, acceleration, and value linearity error between facsimile signature and imitation signature handwriting [11]. The Chinese scholars Zeng and Wang pointed out that the pressure of the pen tip or finger should be used when using the resistive electronic signature board for electronic signature. If the pressure is small during writing, the pen will be broken or unable to cross, and the handwriting and strokes will be stiff [12]. Wang and Wang pointed out that the technical principles of capacitive and resistive electronic signature boards are different. As long as they contact charged objects, they can form electronic signatures without pressure. The generated electronic signature handwriting is also relatively coherent, and the overall handwriting feature effect is ideal [13]. Zheng et al. believed that the electronic signature generated by the electronic signature has high similarity compared with the traditional study and pen written signature. The usage of electronic signature handwriting can accurately capture the writer's everyday writing habits, such as stroke crossing characteristics, continuous stroke characteristics, and handwriting structure features, which will not be affected by other instruments. Apart from it, these characteristics of the potential writers play a significant role in describing the nature of a writer or simply how to differentiate writing of one author from the other with expected accuracy [14].

RETRACTED

## 3. Computer Vision Technology

Computer vision is an artificial intelligence field that teaches computers to interpret and comprehend images. Machines can properly recognize and classify objects using digital images from cameras and movies, as well as deep learning models, and then react to what they “see.” Or simply, we can define it that it is a field of computer science where the main theme is to enable the computer or robots or any other electronic device to perceive things just as human beings do in the real world. In this regard, various approaches have been reported in the literature, but it is still an open research domain.

### 3.1. Visual Tracking Method

Visual tracking can accurately identify the moving target in the image sequence and obtain the basic motion parameters such as speed, pose, motion trajectory, and acceleration of the moving target. Usually, an ideal visual tracking system must have the basic characteristics of real-time, accuracy, and robustness. However, there are still many problems in the real environment. When projecting a three-dimensional image onto a two-dimensional image, there will be information loss, scaling, rotation, and displacement of the target in the scene, and it will also be affected by noise, illumination change, and occlusion in the background environment. Various academics have proposed solutions to this challenge, resulting in a tracking algorithm that is becoming increasingly diverse and flawless. The data-driven tracking method is the most extensively used of these approaches. The optical flow method is a good example of this approach. This method has been extensively utilized in various domains due to its overwhelming characteristics.

If the velocity vector is assigned to each point on the two-dimensional motion scene, it can represent the motion speed, direction, and distance. Optical flow method is a motion analysis method based on this assumption, which can analyze the image changes caused by motion interference in each interval. The optical flow field represents the velocity field on the three-dimensional motion of the target point. When using this method, it should first assume that the gray value on the target is fixed, and the adjacent points move in the image plane in a similar way.  Figure 1 shows the calculation flow of the optical flow method.

Next, select time *t*+*δt* and time *t* to calculate the pixel position motion, assuming that the pixel point of *I* (*x*, *y*, *t*) gray value is (*x*, *y*, *t*), and the motion mode of the two image frames is *δx*, *δy*, *δt*. The image constraint is calculated from the following equation:

(1) $$\begin{array}{c} t+\delta t\delta x\delta y\delta \\ I\left(x,y,t\right)=I\left(x+\delta x,y+\delta y,t+\delta t\right). \end{array}$$

If the motion is small, Taylor expansion at *I* (*x*, *y*, *t*) position can be selected to obtain the following results after taking out all the higher-order terms:

(2) $$\begin{array}{c} I\left(x+\delta x,y+\delta y,t+\delta t\right)=I\left(x,y,t\right)+\frac{\partial I}{\partial x}\partial x+\frac{\partial I}{\partial y}\partial y+\frac{\partial I}{\partial t}\partial t+\cdots . \end{array}$$

After simultaneous calculation of the above two formulas, the following formula is obtained:

(3) $$\begin{array}{c} \frac{\partial I}{\partial x}\partial x+\frac{\partial I}{\partial y}\partial y+\frac{\partial I}{\partial t}\partial t=0. \end{array}$$

Furthermore, draw

(4) $$\begin{array}{c} \frac{\partial I}{\partial x}Vx+\frac{\partial I}{\partial y}Vy+\frac{\partial I}{\partial t}Vt=0. \end{array}$$

The above formula is that, in the optical flow constraint equation, *V*_*x*_ is the *I* (*x*, *y*, *t*) streamer in the *x* direction, and *V*_*y*_ is the *I* (*x*, *y*, *t*) streamer in the *y* direction. Rewrite the above formula as

(5) $$\begin{array}{c} I_{x}V_{x}+I_{y}V_{y}=-I_{t}. \end{array}$$

The advantage of optical flow method is that it does not need to predict the scene information. It is widely used in computer vision and pattern recognition.

RETRACTED

### 3.2. Motion Modeling and Tracking Algorithm

Kalman filtering is an algorithm for estimating unknown variables based on measurements collected over time. Kalman filters have proven to be effective in a variety of applications. Kalman filters are simple in design and need little processing power. Likewise, Kalman filter has been defined as minimum variance estimation applied in time domain. However, based on Hidden Markov model and linear algebra, the dynamic system is represented by Markov chain, and the system is constructed on the linear operator disturbed by Gaussian noise. The running state of the system is represented by the vector based on the real number of elements.

Define the matrix for each step *k*, or define Bk. The circle represents the vector relaxation matrix, while the asterisk is Gaussian noise, and the lower right side identifies the covariance matrix. The estimated state *X*_k_ without input at *t*_k_ is explained by the following formula:

(6) $$\begin{array}{c} X_{k}=\Phi_{k,k-1}X_{k-1}+\Gamma_{k-1}W_{k-1}. \end{array}$$

The measurement of *Z*_k_ is described by the following formula:

(7) $$\begin{array}{c} Z_{k}=H_{k}X_{k}+V_{k}. \end{array}$$

*H*_k_ is the measure matrix in the formula above. Φ_*k*,*k*−1_ represents the transfer matrix, Γ_*k*−1_ represents the system noise excitation, *V*_k_ represents the observed noise matrix, and both *V*_k_ and *W*_k_ meet the following formula requirements:

(8) $$\begin{array}{c} \left.\begin{array}{c} W\left[W_{k}\right]=0,Cov\left[W_{k},W_{j}\right]=E\left[W_{k},W_{j}^{T}\right]=Q_{k}\delta_{kj},\\ W\left[V_{k}\right]=0,Cov\left[V_{k},V_{j}\right]=E\left[V_{k},V_{j}^{T}\right]=R_{k}\delta_{kj},\\ Cov\left[W_{k},V_{j}\right]=E\left[W_{k},{}_{V}^{j}\right]=0. \end{array}\right\} \end{array}$$

The above *Q*_k_ denotes the noise variance matrix, and *R*_k_ denotes the measurement matrix. If *Z*_k_, *X*_k_, *V*_k_, *Q*_k_, *W*_k_, *R*_k_ can meet the requirements of the Kalman state and Bayesian estimation criteria, the discrete Kalman filter equation is described below.

RETRACTED

First, predicting the state at *k* − 1 time:

(9) $$\begin{array}{c} {\hat{X}}_{k/k-1}=\Phi_{k,k-1}{\hat{X}}_{k-1}. \end{array}$$

Second, state estimation:

(10) $$\begin{array}{c} {\hat{X}}_{k}={\hat{X}}_{k/k-1}+K_{k}\left(Z_{k}-H_{k}{\hat{X}}_{k/k-1}\right). \end{array}$$

Finally, filter gain:

(11) $$\begin{array}{c} K_{k}=P_{k/k-1}H_{k}^{T}\left(H_{k}P_{k/k-1}H_{k}^{T}+R_{k}\right)-1. \end{array}$$

$\hat{X}k$ (*k* = 1,2, ...) is recursively obtained after initialization. The state estimation algorithm uses iterative recursive inference theory to update alternately and is suitable for computers.

## 4. Dynamic Characteristics of Electronic Signature and Conventional Signature Handwriting Based on Computer Visual Technology

In this study, people's conventional signature handwriting and electronic signature are selected as the main research objects during the process of comparing and analyzing the dynamic characteristics of electronic signature and conventional signature handwriting based on computer vision technology, and the dynamic characteristics of user's handwriting on electronic signature are extracted using electronic signature equipment and analysis software [15]. Under the same conditions, the dynamic properties of a person's traditional signature and electronic signature handwriting are studied experimentally. The challenges that affect the dynamic characteristics of electronic signature handwriting are evaluated after changing the conditions to analyze the dynamic differences between traditional signature and electronic signature handwriting.

At present, most of the components of electronic signature devices are digital pens and screens. Today in the market, the working principle is used to classify the types of digital screens as capacitive, electromagnetic, and resistance screens [16]. The technology used on the electromagnetic screen is electromagnetic induction, which is used to write with the electromagnetic pen. Capacitive screen uses human current induction technology. Users can write directly with their fingers without using an electromagnetic pen. The essence of resistance screen is a sensor, which works by using the principle of pressure induction, using a normal digital pen. Electromagnetic screens are widely used in organizations, units, and enterprises. There are few capacitive screens on the market, and resistance screens have been eliminated. In this study, the electronic signature device manufactured by Wacom Company is selected, and its appearance is shown in Figure 2:

After collecting the user's electronic signature handwriting through the electronic signature device, the dynamic feature data can be obtained, and the collected data can be analyzed by the parsing software, using MovalyzeR software to parse the original data on the dynamic characteristics of the electronic signature track.

RETRACTED

### 4.1. Dynamic Feature Extraction

#### 4.1.1. Writing Average Speed, Time Length, and Average Pressure Characteristics

This feature is the time, average pressure, and average speed required for electronic screen contact, electromagnet pen, or regular writing to play signature. The unit is *t*, cm.s^−1^, m/s. The speed and time are recorded true values, and the pressure is expressed by the pressure level and belongs to the virtual value.

#### 4.1.2. Characteristic of Writing Speed Variation Curve and Pressure Distribution

Whether people sign on paper or on an electronic screen, the parameters such as writing pressure and speed are not fixed. They adjust their weights based on sitting position or pen, which should be studied in conjunction with the theory of handwriting verification. At the same time, changes in stress and speed during writing also indicate changes in writing habits. Thus, changes in writing speed can be expressed by the rhythm of writing and are strongly related to time. There is a strong correlation between pen strength and signature position according to the change of writing pressure. Therefore, in this study, when comparing the dynamic characteristics of conventional signature handwriting with electronic signature handwriting, we need to dig the pressure, speed, and other characteristics information and analyze their dynamic characteristics by combining coordinate location and time.

#### 4.1.3. Obtaining Dynamic Feature Raw Data

This study uses electronic signature, which has already been defined in the above sections, equipment, and parsing software to collect the original data of the user's handwriting dynamic characteristics on electronic signature, which contains the average writing speed, length, average pressure of the user and the coordinates, serial number, speed, and pressure values corresponding to each signature track [17]. In this study, 10 subjects aged 20–28 years were selected for the study. Data on average speed, writing duration, and stress characteristics of electronic signatures and conventional signatures were collected from 10 participants, which are given in Table 1:

In the process of writing an electronic signature track, the electronic signature device records the motion track of the electromagnetic pen in a series of points. The essence of the electronic signature track is to connect a series of locations with equal time intervals, which is shown in Figure 3.

The electronic signature device keeps records of coordinates, numbers, speeds, and pressure values of all the positions on the electronic signature handwriting in order before and after use. It is important to note that the sequence number is predominantly used in the literature as well as in this study to describe more specifically and efficiently the duration of the signature. The sequence number is the order of the sites formed and serves as an important basis for the calculation of the signature duration [18, 19]. In this study, one of the 10 experimenters was randomly selected, and the coordinates, serial numbers, pressure, and speed values at each location were listed in Table 2. The sampling device selected here has a frequency of 200 Hz, and 200 loci can be saved in one second.

RETRACTED

### 4.2. Experimental Data Analysis Method

#### 4.2.1. Time Series Similarity Measurement and Analysis

When analyzing the similarity measurement of time series, this study extracts the velocity value and sequence number of each site on the signature track, first converts the sequence number into time, represents it on the abscissa, and the ordinate is the velocity value, so as to complete the writing velocity curve of electronic signature and conventional signature. By analyzing the change curve of signature writing speed, the characteristics in the graph mainly include the number, position, and value of peaks, so the peaks should be extracted.

#### 4.2.2. Dynamic Time warping (DTW)

Dynamic time warping is a time series analysis algorithm for determining the similarity of two temporal sequences that may vary in pace. Dynamic time warping is a versatile technique that can be used in a variety of settings. It is easy to recognize examples of dynamic temporal warping's uses in everyday life, as well as its fascinating future applications, once you comprehend the concept. Among the multiple handwriting signatures written by the same person under the same conditions, it is impossible to write at the same speed and time. Therefore, the length of the peak curve of speed change is also different. For the curve with small peak position offset but very similar shape, if the correlation coefficient is calculated, the result will be reduced. Here, the dynamic time warping algorithm (DTW) is introduced into the analysis.

DTW algorithm can align two random curves according to the “maximum similarity principle,” so as to better calculate the correlation coefficient and avoid the problem contrary to the above facts [20]. The following is the basic principle of DTW algorithm:

Let *C* and *Q* be two different curves, and their lengths correspond to *m*, *n*, *Q* = *q*_1_, *q*_2_, ..., *q*_*j*_,..., *q*_*n*_; *C* = *c*_1_, *c*_2_, ..., *c*_*j*_, ..., *c*_*m*_; *n* is not equal to *m* at the same time. By creating *n* × *m* matrix, assuming that the (*i*, *y*) matrix element is the Euclidean distance between *c*_j_ and *q*_*i*_, which can be expressed as *d* (*q*_*i*_, *c*_*j*_), *d* (*q*_*i*_, *c*_*j*_), *d*(*q*_*i*_, *c*_*j*_)=(*q*_*i*_ − *c*_*j*_)^2^, which is expressed by the alignment of *c*_j_ and *q*_i_ by (*i*, *y*) matrix. Multiple point paths on this matrix are obtained through DP algorithm. The points passing through are the aligned points on the two curves, and this path is a *W*-regular path. Assuming that the k-th elements on W are represented by *w*_*k*_ = (*i*, *j*)*k*, the mapping of *C* and *W* curves is defined as *W* = *w*_1_,*w*_2_,...,*w*_*k*_,...,*w*_*k*_, max (*m*, *n*)≤*K* < *m* + n − 1. By combining monotonicity constraints and continuity constraints, the following is the path with the lowest cost of regularization investment:

(12) $$\begin{array}{c} \text{DTW}\left(Q,C\right)=\min\left\{\sqrt{\sum_{k=1}^{k}\frac{w_{k}}{K}}\right\}. \end{array}$$

The *K* at the denominator position in the formula is used to compensate the regular paths with different lengths. It can be seen that the two curves with the shortest distance are removed, and the shape similarity is high.

RETRACTED

## 5. Comparison and Analysis of Dynamic Characteristics between Electronic Signature and Conventional Signature Handwriting

### 5.1. Analysis of Writing Duration Characteristics

When analyzing the characteristics of writing duration, this study selects the average writing duration of electronic signature and conventional signature of 10 experimenters and draws the following broken line diagram according to this value, as shown in Figure 4.

Analyze and compare the writing time of electronic signature and conventional signature shown in Figure 4. The writing time of electronic signature is longer than that of ordinary conventional signature. The time of electronic signature of most participants is basically the same as that of conventional signature, and only some people are longer. The main reason is that some people are not familiar with the way of electronic signature and worry that the wrong writing cannot be modified, so they prolong the writing time. Additionally, some people are very eager about accuracy, and this is the main reason behind the extra time needed by various or potential class of writers.

### 5.2. Average Velocity Characteristic Analysis

When analyzing the signature average speed characteristics, this study selects 10 experimenters to analyze the signature average speed. According to the obtained test results, draw the following comparison between the average speed of electronic signature and conventional signature handwriting, which is shown in Figure 5.

RETRACTED

According to the analysis of the comparison results of the average speed of electronic signature and conventional signature handwriting shown in Figure 5, the average speed of electronic signature and conventional signature of the vast majority of participants is basically the same, with great differences among very few people, and it is generally shown that the average speed of conventional signature handwriting is higher than that of electronic signature, and the average speed of each person fluctuates greatly, which is related to each individual participating in the experiment.

### 5.3. Average Pressure Characteristic Analysis

When analyzing the average pressure characteristics, this study selects the average pressure data of electronic signature and conventional signature handwriting of 10 experimenters, collects the average pressure data through the equipment for analysis, and draws the broken line diagram of the comparison of the average pressure of electronic signature and conventional signature handwriting, as shown in Figure 6.

Figure 6 shows the average pressure results of electronic signature and conventional signature handwriting of 10 experimenters. The relevant information can be mastered after the analysis of broken line diagram. The results show that the average pressure of conventional signature is higher than that of electronic signature. Because some people worry that too much pressure will damage the equipment when using electronic signature, the average pressure of electronic signature is lower than that of conventional signature.

### 5.4. Comparative Analysis of Dynamic Characteristics of Handwriting

Through the experimental analysis of this study, it is concluded that, compared with the ordinary signature handwriting, the electronic signature handwriting written by a person on the electronic equipment has strong stability in font shape, overall style, font inclination, special writing method, and stroke order. There are some changes in the characteristics of pen movement, layout, stroke matching, and connectivity, which are reflected in the dragging of pen collection, scattered layout, bending and shaking of strokes, and the change of stroke matching. Among them, the most obvious changes are the handwriting size, writing level, and writing trace. In this aspect, the font becomes larger, the writing level decreases, and the handwriting characteristics weaken. The occurrence degree and probability of the above characteristics are different in the research process. By counting the occurrence probability of different handwriting change characteristics, the comparison is given in Table 3.

RETRACTED

## 6. Conclusion

In recent years, with the rapid development of e-commerce industry, all kinds of handwriting input devices are also widely used in various fields and have become a common way of signature in people's life. This study analyzes the collected dynamic characteristic data of traditional signature and electronic signature handwriting based on computer vision technology, which is convenient for the effective development of identification work, can realize the scientific inspection of electronic handwriting, and can speed up the rapid development of handwriting inspection discipline. There is a significant difference between electronic signature handwriting and regular signature handwriting, which differs significantly in terms of electronic signature equipment, signature content, and user signing habits, as well as the end product. Apart from it, we have tried to compare the handwriting differences between electronic signature and conventional signature from three aspects, writing time characteristics, average speed characteristics, and average pressure characteristics, which is helpful in improving the accuracy of electronic signature.

## Figures and Tables

**Figure 1:** Calculation flow of the optical flow method.

**Figure 2:** Electronic signature device.

**Figure 3:** Location map of handwriting.

**Figure 4:** Comparison of writing time between electronic signature and conventional signature.

**Figure 5:** Comparison of average handwriting speed between electronic signature and conventional signature.

**Figure 6:** Comparison of average handwriting pressure between electronic signature and conventional signature.

**Table 1:** Electronic signature handwriting duration, average speed, and average pressure.

Order (time)	The writing time (s)	The average velocity (cm·s^−1^)	Average pressure (stage)
1	8.83	3.12	324.1
2	7.65	3.47	308.6
3	7.49	3.51	302.1
4	7.53	3.56	303.5
5	7.83	3.36	308.5
6	8.59	3.38	316.6
7	8.09	3.34	319.9
8	8.19	3.36	326.3
9	8.37	3.37	323.9
10	7.83	3.35	332.7

**Table 2:** Signature handwriting position serial number, coordinates, speed value, and pressure value.

Number	*X* (cm)	*Y* (cm)	Pressure value (level)	Speed value (cm·s^−1^)
1	6.32	6.06	153.0	0.28
2	6.32	6.06	212.5	0.23
3	6.32	6.06	239.3	0.25
...	...	...	...	...
10086	9.69	5.26	23.7	6.47

**Table 3:** Comparison of dynamic characteristics between electronic signature handwriting and ordinary signature handwriting.

Handwriting feature type	Changes in signature morphology	The number of (30)	Proportion (%)
Character of writing level	Decline in writing	23	73.4
Layout characteristics	Adjust word combinations	13	41
Font character	--	0	0
The slant of a word	--	0	0
Strokes match and connect	Change the collocation	15	46.9
Characteristics of words	--	0	0

RETRACTED

## Data Availability

The datasets used and/or analyzed during the current study are available from the corresponding author upon request.
